The article "Innovative Design of Intelligent Health Equipment for Helping the Blind in Smart City" was retracted in 2023. Reasons: signs of a paper mill; suspected computer-generated content; unreliable results or conclusions; concerns about the data.

# Innovative Design of Intelligent Health Equipment for Helping the Blind in Smart City

**DOI:** 10.1155/2022/3193193

**Published:** 2022-07-08

**Authors:** Chang Wei, Lv Guang, Liu Bin, Ruoxi Li

**Affiliations:** ^1^School of Arts and Media, Suqian University, Suqian, China; ^2^School of Foreign Studies, Suqian University, Suqian, China; ^3^Fujian University of Technology, Fuzhou, Fujian, China

## Abstract

The rapid advancement of information technology in today's modern society is contributing to an increase in the general degree of civilization in society. People are pleased with technological progress, but they are also becoming more aware that a major challenge confronting the advancement of social civilization at the moment is determining how to alleviate the difficulties associated with traveling and participating in social activities for the blind, as well as increasing the frequency with which they go out, travel, and participate in other activities. The blindness equipment that is now accessible in China is no longer suitable to meet the needs of blind people, but the growth of smart cities offers an opportunity to change this. Guide devices are crucial among the numerous types of equipment to assist the blind, and in order to better fulfill their various demands, we must upgrade and optimize the existing devices. The Chinese People's Daily highlights some of the key barriers to blind people's access in its 2019 article: random parking that blocks blind lanes; and “snake” and “broken” blind lanes that are not created with blind people's access in mind. In a smart city, accurate placement via smart maps helps alleviate a number of traffic-related issues for blind individuals. In this paper, we propose an intelligent guide device and interactive software to provide a more intelligent way for blind people to travel, which can effectively improve blind people's traffic conditions and make their travel easy, convenient, and safe, reflecting society's concern for blind people.

## 1. Introduction

IBM introduced “Smart Planet” for the first time in November 2008. In today's world, with the fast growth of society, economics, and information technology, smart cities unavoidably arise in the process of urbanization in nations all over the world. Ensuring livable circumstances within the backdrop of such fast urban population increase worldwide demands a greater grasp of the smart city idea. The urgency around these concerns is pushing many cities across the world to discover wiser methods to manage them. These cities are increasingly labeled with the name smart city. One approach to imagine a smart city is as a symbol of a sustainable and livable city [1]. The most fascinating part about smart cities is its development possibility and operating manner. Their objective is not merely to be intelligent, but to accomplish intelligent management of cities by scientific analysis of urban development data so that urbanization becomes more ideal and sustainable. At the same time, the rapid development of 5G information technology provides not only a more realistic environment for the deepening of multithing interconnection in smart cities, but it also makes this environment available. 5G and developing technologies like artificial intelligence will continue to change, which will open up new opportunities for building and developing information and digital systems in the business of helping people with disabilities.

The article "Innovative Design of Intelligent Health Equipment for Helping the Blind in Smart City" was retracted in 2023. Reasons: signs of a paper mill; suspected computer-generated content; unreliable results or conclusions; concerns about the data.

According to statistics, there were 134.1 billion people and 8.24 million blind people in 2010; as of 2018, the country has increased to 139.5 billion and the number of blind people has exceeded 17 million; that is, in 2010, there was 1 blind person for every 162 blind people, and in 2018, it reached 82. That means there are about 140 million people in the world with bad eyesight, and 75% of them, or more than 100 million, cannot fix or improve their eyesight without surgery or diopter correction. Still, 25% of people with poor eyesight need low vision treatment, such as using low vision equipment and visual rehabilitation instruments [2]. However, so many blind people are hard to see in their everyday lives, partly because of their limited access to transportation. With the creation of smart cities in China, notably the growth of technology and information technology, ideal conditions have been established to improve traffic safety for the blind. A blind person is a visually challenged individual in a world where they can only perceive the world via their sense of touch and hearing. Solving the challenges of travel difficulties of blind people, enhancing their travel, travel rate, and participation in social activities is an important issue in advancing the creation of social civilization in China at now.

With the construction of smart cities and networks, blindness devices and blindness software are constantly being upgraded, and the development of technology is simultaneously changing the way of life of blind people. The general environment in which partially sighted people live is also gradually becoming intelligent. To understand the dynamic life of blind friends in real time through guide devices, it is necessary to transform the guide stick with technological innovation.

Even if accessible devices were installed throughout a city or area, this would not guarantee that people who are partly sighted would have adequate mobility or that their transportation requirements would be met. In this article, we conducted a survey on accessibility and a comprehensive investigation of the findings. We discovered that urban roads are indeed difficult for the blind and that since upgrading the existing guide canes with contemporary information technology and advanced technical means can be a good solution to the current problems, this will greatly improve the safety and convenience of transportation for the blind, and this will promote the development of a harmonious society. A way of thinking is merely one aspect of design. It is also a human collective process that is molded by history, culture, and the rules of society or organizations [3].

The article "Innovative Design of Intelligent Health Equipment for Helping the Blind in Smart City" was retracted in 2023. Reasons: signs of a paper mill; suspected computer-generated content; unreliable results or conclusions; concerns about the data.

Based on the idea of barrier-free design, the design is based on the background of smart city; combined with the current needs of blind people outwardly; analyzed and reasonably screened out the attributes and functions required by the city and blind people to adapt to the requirements of the city and blind people, using a variety of expertise and technologies; and reasonably selected and used materials to systematically solve the overall quality and structure, obstacle avoidance, and accessibility for blind people. Additionally, the project intends to design a service robot that can be used in exhibitions, as well as provide a management and dispatching system as well as a remote cinematic reality system. This system will have both autonomous reception functions and a panoramic visual and voice system, and it will be able to be controlled through the use of panoramic reality interaction. This research looks at new electronic travel aids for people who are blind or have trouble seeing. For this group, the white cane is still the most common tool [4].

The project aims to improve the traffic conditions of blind people by providing accurate map positioning on the basis of smart city, and solving a series of problems faced by blind people in traffic through the combination of APPs and devices to help blind people.

## 2. Research Status: Development of Blind Guide Sticks and Guide Software

### 2.1. The Concept of a Smart City

IBM first suggested the idea of a “Smarter Planet” in November of 2008, and since then, the company has been working on a worldwide program called “Smart City.” The fundamental model of a smart city can be summed up as follows: making full use of advanced information technology; interconnecting multiple things with the Internet of Things; relying on cloud computing; using an intelligent mobile terminal big data analysis platform for data analysis; through monitoring, analysis, integration, and intelligent response; integrated functions of various departments from all walks of life; joining hands to open a smooth interconnection channel; and opting for integration and opting for intelligent response. During the process of accelerated urbanization, which is frequently accompanied by population growth, housing tension, environmental damage, traffic congestion, and other types of “urban diseases,” in order to deal with such problems, to promote the healthy, safe, and sustainable development of cities, the development of “smart cities” has become a common requirement and trend for the development of countries all over the world. This is because the development of “smart cities” can help deal with population growth, housing tension, environmental damage, and traffic congestion, and China has emerged as one of the most important locations for the development of smart cities at a time when building of smart cities all over the world is experiencing a surge. In this article, we will provide a high-level overview of the fundamental elements that make up a smart city, which we will define as a city in which information and communication technology (ICT) is combined with traditional infrastructures, coordinated, and integrated with the help of new digital technologies [5].

The article "Innovative Design of Intelligent Health Equipment for Helping the Blind in Smart City" was retracted in 2023. Reasons: signs of a paper mill; suspected computer-generated content; unreliable results or conclusions; concerns about the data.

As of June 2016, 95 percent of cities above the subprovincial level and over 76 percent of prefecture-level cities across the country, for a total of over 500 cities (more than half of the total number of smart cities created in the world, including all urban spatial forms and scales), have explicitly proposed or are building chase cities in the annual government work reports, and China has become the main testing ground for the creation of smart cities in the rest of the world, with a focus on urbanization and technological advancement. The experience gained over the course of the previous five years demonstrates that megacities are the primary targets of China's smart city industry in order to achieve considerable advancement and have replicable results.

### 2.2. The Significance of Smart Blindness Aids in Smart Cities

According to the World Health Organization (WHO) and the Second China Disability Survey (2006), the number of blind persons in China has risen to 12.33 million, accounting for 20% of the global blind population. People who are visually blind can navigate unfamiliar situations with the assistance of other people, canes, or guide dogs that have undergone specific training. Guide dogs can provide their owners with the most mobility and independence imaginable, but training these dogs can be costly, and selective breeding is required [6]. Despite the fact that there are many accessible facilities for the blind (such as blind alleys and sound crossing), they are insufficient to meet the demands of the blind. Blind people's daily lives are made more difficult by their inability to see, especially as city roadways become more complex and the number of vehicles increases. When formerly marginalized people with dementia gain access to the same social resources and chances for involvement as the general community, they demonstrate a greater level of social and cultural development. As a result, the question of how to ensure that blind people can travel safely has developed as an important research topic in our country in modern culture. The term “smart cities” is defined as “providing a better urban life for human beings by sensing, analyzing, and integrating various types of important information about the operation of the city and responding intelligently to various needs of people's livelihood, environmental protection, public safety, urban services, industrial and commercial activities, and so on” in IBM's book “Smart Cities in China.” The growth and formation of smart cities has created a chance to address this issue, which is defined as “creating a better environment.” The goal is to make effective use of modern information technology to run and manage the numerous guiding devices. Because of China's continued development in the field of intelligent interaction, as well as the ongoing development of related technologies, there is already some opportunity for the building of guide equipment and guide software suited for the blind to travel securely. Furthermore, many issues, such as difficult travel and travel challenges, are common throughout the creation and building of smart cities. There is one blind person for every 82 blind individuals on average, and the number of blind persons in China accounts for 20% of the total number of blind people worldwide, the highest percentage in the world. According to data, the overall population of the country reached 1.395 billion in 2018, including 17 million blind individuals. The most major impediments are visual impairment and loss of eyesight, followed by traffic congestion in cities; specialized services for the blind, such as blind corridors and auditory notifications for crossing the street, do not sufficiently meet the needs of blind people. Blind persons are a socially disenfranchised minority, but they have access to the same social resources and chances for social participation as other disabled people. Furthermore, the proportion of blind individuals who go out, travel, and engage in social activities has increased, which is an important measure of a modern society. As a result, finding answers to the mobility challenges faced by the blind has attracted the attention of people all over the world, and it is now one of the most crucial concerns confronting attempts to improve human civilization. The goal of this study was to illustrate the research that went into the development of a breakthrough travel equipment that facilitates independent movement for blind or elderly passengers. This support will be provided using geographical information systems (GIS) and the global positioning system (GPS) technologies [7, 8].

The article "Innovative Design of Intelligent Health Equipment for Helping the Blind in Smart City" was retracted in 2023. Reasons: signs of a paper mill; suspected computer-generated content; unreliable results or conclusions; concerns about the data.

When developing a new and reliable navigation system, it is essential to take into account both the goals that are to be accomplished as well as the technology that will be utilized. The real-time assistance prototype machine utilizes the principle of object detection in its operation. The following three significant questions are investigated: “what to detect,” “how to monitor,” and “how to portray the information that has been discovered” [9].

As product design students and aspiring designers, we should have a strong sense of social mission and duty, and good design may directly contribute to the development of people's material and cultural life in a variety of ways. This project intends to improve blind people's travel experiences by assisting visually impaired individuals through the use of technologies such as GPS and Bluetooth, as well as accomplishing the interconnection of things through the interaction between the product and the guide software. As a result, persons who are blind will be able to travel in a more intelligent and easy manner.

### 2.3. The Development Status of Blindness

#### 2.3.1. Development Status of the Blind Cane

As social science advances, the general public is becoming more aware of the difficulties that visually impaired people confront in their daily lives. As a result, several travel guidance gadgets and systems are currently being investigated and developed as potential answers to the challenges that visually impaired persons experience on a daily basis. The guiding devices that have been developed to date might be classified as handheld, wearable, or mobile devices. According to the American Foundation for the Blind, the objective of any sensory aid is “... to detect and identify items and give information that allows the user to establish (within acceptable tolerances) the range, direction, size, and height of objects.” It enables noncontact following and tracking, allowing the traveler to acquire directional cues from physical structures in strategic locations in the surroundings, with further object identification if possible [10].

The handheld guide is a new type of guide that is based on the electronic guide stick. It was developed by a domestic and foreign expert based on the ultrasonic distance measuring principle, and it has a wide range of detection, making it capable of detecting road obstacles, road bumps, and other types of information. It is not feasible to engage in any form of social activity or walk outside if one does not own the necessary instruments. Canes of white color and dogs trained to assist the visually impaired are the most often used aids [11]. The fact that it is unable to navigate is its most significant drawback; nevertheless, because it may be integrated with other navigation systems, it can be used to assist blind persons more effectively when traveling. Because blind perception technology does not require any information, it possesses the benefits of having a high recognition success rate, quick perception time, simple operation, and straightforward implementation, and as a result, it has the potential to be used in a variety of contexts. Blind people make up a distinct category in society, and as such, society owes it to them to provide them with greater care and attention, making it possible for them to lead more independent lives [12]. Nevertheless, the most significant challenge is determining how risky a life of blindness can be [13]. Traditional navigation instruments are largely blind canes; blind individuals detect direction by tapping the ground or wandering around an object. The structure is simple, with a single purpose, and it is simple to use; yet, the secondary effect is not clear. In reality, when using the blind, blind people will encounter numerous issues such as poor road conditions, uneven terrain, and hanging in front of barriers; regular canes cannot be proven correct, which has a substantial negative influence on the safety of blind travelers [14].

The article "Innovative Design of Intelligent Health Equipment for Helping the Blind in Smart City" was retracted in 2023. Reasons: signs of a paper mill; suspected computer-generated content; unreliable results or conclusions; concerns about the data.

Wearable guide devices are less prevalent than electronic guide canes, which frequently include CDM-I type guide glasses. These gadgets are typically guide glasses that are similar to electronic guide canes. Two ultrasonic sensors and an earphone device deliver reflected ultrapulse waves to the front of the spectacles. The blind individual may perceive barriers in front of them based on changes in the earpiece of the glasses they wear. Existing research must be examined historically, beginning with the first studies on electronic travel aids and extending all the way up to the use of modern artificial vision models for BVIP navigation. This analysis will be required. A variety of devices have been proposed for navigating BVIPs, including an electronic cane or guide dog, an infrared-based cane, a laser-based walker, and many others. However, the bulk of these systems have limitations, such as infrared and ultrasonic-based aid having limited capacities for object recognition at short ranges [15].

On the other hand, mobile guides are far less common. These are mostly guide robots that can take people to the road, assess their surroundings as they walk, and identify various types of traffic indicators such as crosswalks and traffic signals [16].

There are already some navigation products available on the market for the blind, particularly for wearing and moving around. One example of this is the Aira glasses, which were developed by Kanuganti Suman and his research team at the University of California, San Diego. These glasses are similar to a blind person's third eye, but they are unable to “see” the real world. The Aira glasses function similarly to the third eye of a blind person; however, the wearer is unable to “see” the actual world and can only communicate with the “Aira helper” standing behind them through a camera located in the middle of the Aira spectacles. It is thought that external light sources will have a direct impact on the quality of the picture, which will in turn have an impact on the visual effect. This belief stems from the expensive cost of optical guides (see Figure 1).

#### 2.3.2. Development Status and Trend of Blind Guidance Software

People who are blind or have a vision impairment sometimes face difficulties while attempting to move around alone. Mobile devices, such as smartphones, have been the source of ground-breaking innovations in recent years [17]. These devices serve as handy platforms for the delivery of assistive technology in the form of mobile applications. Additionally, disability programs have been impacted by the fast development of both the hardware and software for cellphones. As can be seen in Figure 1, the mainstream app store already offers a variety of interactive software options for those who are visually impaired. The “Visible ICanSee” app is a communication and social app that was designed by Xing Sun, an independent app developer. Its purpose is to assist those who are visually impaired and it is split into two different ports: one for those who are visually impaired and one for those who volunteer to assist them. The position of the visually impaired individual is matched with that of the volunteer, and the system then guides the volunteer toward the person who need assistance. There is a community for the visually impaired within the “Visible” app. Within this community, volunteers and individuals who are visually impaired may make friends and chat to one other, and they can also provide assistance to those who are blind from a spiritual standpoint.

The article "Innovative Design of Intelligent Health Equipment for Helping the Blind in Smart City" was retracted in 2023. Reasons: signs of a paper mill; suspected computer-generated content; unreliable results or conclusions; concerns about the data.

The “Ember” app from Changchun Yunhai Technology is dedicated to creating a barrier-free living service platform for the blind, aiming to provide comprehensive, multifaceted, and in-depth services for the blind to enhance their well-being. The main function of the app is to link the studio's smart glasses for the visually impaired with the app so that the smart glasses can identify objects around them and other functions to achieve accessibility for the blind.

However, they focused on the difficulties of the blind when they designed the software to help them go out, and did not completely abandon the stereotypical view of the able-bodied toward the blind, providing functions that are not rigidly needed by the visually impaired and lacking in functionality. At the same time, the high price of these apps with devices is also a very big obstacle on the road to their popularity.

### 2.4. Development Trend of Blindness Aids

The existing problem of urban blind guidance equipment has been very serious; with the development of society, it will inevitably put forward new development requirements, and the new type of blind guidance equipment should be developed toward the following two aspects.

#### 2.4.1. Intelligent (Interactive) Design

The traditional guide cane, with its single function, has not been as effective as it could be. Thanks to the rapid development of computer vision and sound recognition technology, current aids can not only automatically assist users in identifying paths and precisely indicating the orientation of obstacles but also allow for two-way human-machine interaction, allowing users to send service requests to the cane at any time and send signals to the guide software through the cane's Bluetooth connection. However, at present, the rigid guide cane is still limited to individual applications for the blind, and its role is very limited. In the development of smart cities, guide devices are also moving toward intelligence; for example, in this process, people can interact with blind people and their auxiliary guide devices so that they can make better use of these guide aids to achieve better results.

#### 2.4.2. User-Friendly Design

Most of the current guide devices focus only on the needs of basic functions and lack sufficient attention to user experience, comfort, and safety so that many blind people are reluctant to use them, and the devices that have taken a lot of energy and effort have become a decoration. Good equipment must be user-centered and user-friendly. Blind people are a special group, and the comfort and individuality of the guide equipment used for individuals are also important. Adding ergonomic principles to the new guide canes makes the old ones more humane. It is important to focus on in-depth research and analysis of the physical characteristics, behavioral characteristics, and spiritual needs of such people, focusing on the safety of the equipment, the ease of use, and the accuracy in information exchange, so as to establish a set of equipment suitable for use and use by people with disabilities to help the blind.

The article "Innovative Design of Intelligent Health Equipment for Helping the Blind in Smart City" was retracted in 2023. Reasons: signs of a paper mill; suspected computer-generated content; unreliable results or conclusions; concerns about the data.

## 3. Survey Results and Analysis of Problems with the Travel of Visually Impaired Persons

### 3.1. Research and Analysis of Blind Travel Problems

Based on the article “Research on the Construction of Barrier-free Facilities System for Traveling Blind People in Smart Cities” and the research on the existing travel problems of blind people in the society, the basic travel characteristics of blind people and the main problems they face were derived.

1. Based on a survey of the number of trips and difficulties faced by blind people, and combined with the results of interviews, it was found that most blind people have a high number of trips and difficulties in going out, but more fully functional guide canes are expensive and unaffordable for disadvantaged groups; guide dogs are expensive to cultivate and have a limited canine life span; and blind people have a very high chance of encountering danger when traveling alone.
2. Communication problems. Because of their own impairments, blind people first have an inferiority complex, and because they have less contact with the outside world, they tend to have problems communicating with strangers and may even be treated unequally. There are no barrier-free facilities for crossing the street. The blind people are unable to know when to cross the street, and they can easily lose their way in the middle of the street and cannot cross the street independently. Analysis of the radius and destinations of blind people's walking trips. The blind people in the interviews generally reflected that although they often go out, they do not travel far due to their visual impairment; that is, the travel radius is very small and mainly by walking, and many places they want to go have not been visited.
3. There are safety hazards due to the absence of blind lanes, the extremely low utilization rate of blind lanes, and the poor state of maintenance. Currently, blind walkways are the main barrier-free facility for the blind, but surveys show that the utilization rate of blind walkways is very low, with only 4% of blind people using them. Many blind people report that the blind paths are potholed, intermittent, and often occupied, so they prefer to use their blind sticks to navigate the road on the blind paths. Construction occupies roads, traffic “cutoffs”, high traffic safety risks, slow construction progress, irregular construction, dust, and multiple roads excavated at the same time; nonmotorized vehicles occupy roads, business, and other illegal road occupancies; nonmotorized vehicles occupy roads, business, and other illegal road occupancies; and no sidewalks, mixed vehicles, and pedestrians.
4. The emergence of the guide cane has brought a boon to the partially sighted group, but the existing guide cane can only be used as an auxiliary device, or need to travel under supervision, and has not solved the problem of difficult travel for the blind in a real sense.

The article "Innovative Design of Intelligent Health Equipment for Helping the Blind in Smart City" was retracted in 2023. Reasons: signs of a paper mill; suspected computer-generated content; unreliable results or conclusions; concerns about the data.

### 3.2. Analysis and Integration of Blind Travel Problems

The inability to travel completely independent and the high cost of travel are important factors that hinder blind people from traveling, and if we can focus on solving these problems, we can improve the travel rate and the social participation rate of blind people. To summarize, there are several major problems that need to be solved, such as the inability to travel completely independently. On the basis of this information, a novel kind of transportation assistance for the visually impaired is presented as a solution to the problem of traffic discomfort in connection with the overall trend of the development of smart cities. The idea behind the design is to make traveling easier and more pleasant for blind people. Intelligence and humanization are at the core of the concept, and GPS, voice recognition, and radar ultrasonic technology are the primary forms of technical support. The goal of the design is to create a travel aid for the blind that is secure, convenient, and dependable.

## 4. Design and Implementation of Intelligent Blindness Aid Devices

### 4.1. Blindness Aid Device Design and Positioning

This project is designed from the perspective of product design, with the intention of exploring a new path for blind people to travel independently and safely through the combination and improvement of guide products and guide software, and breaking the existing limitations of guiding blind people to their destinations and avoiding “cutoffs” and “snakes”. The new software will be able to provide a new way for blind people to travel independently and safely [18].

In order to meet the needs of intelligent city construction, an intelligent blind cane device is designed to interact human-machine with blindness assistance software through simulation and data detection. Through the implementation of the product and the interaction process, it achieves scientificity, operability, efficiency, and smoothness.

The article "Innovative Design of Intelligent Health Equipment for Helping the Blind in Smart City" was retracted in 2023. Reasons: signs of a paper mill; suspected computer-generated content; unreliable results or conclusions; concerns about the data.

Inspired by the current smart sweeper, we can add a radar device to the bottom of the cane and install pulleys that can move freely through 360°, and the smart cane can be connected to a cell phone through a red button that can achieve multiple links, allowing family members to perform real-time GPS positioning through the network, a guide headset recess on the handle and an overall cane charging pile with magnetic charging, and through Braille buttons. The configuration of the headset can provide functions such as oral orientation, intelligent detection, and retrieval of the cane.

In point of fact, the primary objective of a binaural guiding device is to facilitate the user's ability to track the origin of the sound in the most natural way possible. In order to do this, it is necessary to provide the user with an authentic sensation that is in line with what they would experience in an actual circumstance. In order to provide a more lifelike experience, it is necessary to track the movements of each individual user and adjust the audio rendering accordingly [19].

We design a bone conduction headset associated with the guide cane and a matching navigation map system, as well as a one-touch alarm function. The product uses Bluetooth technology to alert the user through the phone's handle and the vibration of the handle, and also guides the user through voice navigation, GPS, and other means. In addition, the system also provides GPS positioning function, and the user can find the corresponding instrument with a single click on the phone and can provide timely feedback of relevant data, thus reducing the working time of the system (see Figure 2).

### 4.2. Guiding Staff Design Concept Requirements

1. Handle: the handle of the guide cane is ergonomically designed into a streamlined shape, which fits the wrist to the maximum extent and carries out humanized design. The invention combines the red Braille button of the handle with various technologies such as roadblock identifier, electronic GPS navigator for the blind, and instant retrieval of public transportation information. The different presses of the individual buttons have different functions, which can effectively prevent blind people from mistakenly touching and can solve the shortcomings of the current blind guide. It can also communicate with the blind person so that the blind person can transmit and receive information as needed, thus better solving the transportation problem of the blind. It can be used as a guide instrument alone or in conjunction with other auxiliary devices, such as electronic guide headsets, guide robots, and smartphones. This device is simple to develop, easy to transplant, and has a certain degree of intelligence. By updating the existing guide devices, the partially sighted group can “see the light again.”
2. Magnetic charging pile: to make it easier for the blind to operate the intelligent guide rod, the intelligent guide rod should have fast charging and one-handed operation. 5 A to 30 A high current transmission design can meet the needs of fast charging and high current. The current magnetic charging device has a waterproof function, and the female end of the magnetic charging cable can reach dustproof and waterproof (IPX8), thus enhancing the safety of the guide and providing a more intelligent equipment for the partially sighted. The product has the advantages of small size, space-saving, and versatile use and is also suitable for combination in the handle of the guide headset.
3. Pulley, radar device: the use of radar distance measurement above the freely movable pulley, imitating the application of distance measurement radar on the car, depending on how miniaturized and portable, now generally uses the camera that can be achieved, and 120-frame camera can basically measure the more accurate, low price, sufficient supply, sturdy, and resistant to manipulation, in addition to the obstacles ahead, but also need to guide them to find the correct road and route. In addition to the high demand for positioning accuracy, details, and immediate reminders, there are special needs for the blind, such as when pedestrians want to cross the street, they must avoid red lights, pedestrian crossings, or underpasses; when making the selection of roads, they should try to avoid the paths without transportation.

The article "Innovative Design of Intelligent Health Equipment for Helping the Blind in Smart City" was retracted in 2023. Reasons: signs of a paper mill; suspected computer-generated content; unreliable results or conclusions; concerns about the data.

### 4.3. Guidance Headset Design Concept Requirements

The design of the headset for the blind is based on the practical function of the headset, using the weak noise reduction ability of the bone conduction headset, so that when the blind wear it out, they can listen to the voice broadcast and be able to distinguish the various sounds of the environment in time, which will greatly reduce the danger of travel and safely follow the guide to the destination. At the same time, taking into account the special situation of blind people who need to wear headphones for a long time, the shape design and material of the headphones must fit the ear shape, skin-friendly, with various physiological factors of blind people as the core, so that the design of the product is to adapt to different sizes and shapes of the ear, in order to achieve wear not tired ear, in line with the needs of blind people's lives and activities.

With this in mind, the designed headset shape is continuously improved and optimized through continuous practice and research in order to achieve convenience, effectiveness, comfort, safety, etc. In the process of design, the pursuit of function and comfort does not abandon the rules of beauty. It should be based on the first two points to give new qualities to the materials, structure, form, and color of the product, and create products that enable blind people to travel and live more beautifully, rationally, effectively, and safely, with the design aim of improving the convenience and safety of blind people's travel and bringing convenience to their lives.

The article "Innovative Design of Intelligent Health Equipment for Helping the Blind in Smart City" was retracted in 2023. Reasons: signs of a paper mill; suspected computer-generated content; unreliable results or conclusions; concerns about the data.

#### 4.3.1. Bone Conduction Headphones Required

Bone conduction is the process of directly transmitting sound waves in the form of vibrations through the skull.

The mechanism of bone conduction relies on the vibration of the skull to produce sound, while the vibration of the jawbone also causes the skull to vibrate. However, we rarely use our own skull to feel it since the vibration of the skull takes a specific amount of energy, and ordinary sound cannot cause the skull to vibrate except through direct contact with the skull. When compared with standard acoustic transmission systems, bone conduction technology eliminates most of the transmission process, allowing sound to be recovered very clearly in a busy setting and ensuring that sound waves traveling through the air do not annoy others.

It does not impede the ears and instead frees both of them, eliminating the agony associated with having to wear it in the ears for an extended amount of time. Furthermore, it has the ability to successfully prevent a number of health risks caused by headphones, such as ear sweat. As a result, bone conduction headphones are extremely pleasant to wear for lengthy periods of time. Another advantage of opening both ears is that it allows you to wear headphones in potentially dangerous situations. When you wear the headset, your ears will be able to detect changes in the surrounding environment more accurately and provide a more accurate assessment of those changes in real time.

### 4.4. Guided Application Page Design Ideas

This program for the visually impaired is a navigation app, which necessitates a one-of-a-kind interface and functionality in the design of the pages so that blind people may use them freely and without hiccups. The majority of blind people rely on mobile operating systems like iOS or Android to read text on web pages in order to obtain information. Because of this, blind people require an easy-to-use web page that is capable of recognizing the necessary buttons for visually impaired people who still have partial vision, as well as an interface design that is appropriate for visually impaired people and includes a voice announcement at all times during the interaction with the interface. When used for navigation outside, the global positioning system (GPS) is a network of 24 satellites that is operated by the armed forces of the United States of America. It is designed to deliver information about a person's whereabouts virtually everywhere on the planet. Because the satellites offer continuously updated location information regardless of whether or not the pedestrian is moving, navigation devices that are based on GPS are an extremely useful help for orientation [20].

The article "Innovative Design of Intelligent Health Equipment for Helping the Blind in Smart City" was retracted in 2023. Reasons: signs of a paper mill; suspected computer-generated content; unreliable results or conclusions; concerns about the data.

Due to the special nature of the visually impaired group, they will encounter problems when traveling that they cannot handle on their own, so they must seek help from the police and guardians, and they also need to be informed about their situation during the journey. Visually impaired people are less able to collect information compared to ordinary people, so they need to get their location and important markers and signs around them before they can navigate.

### 4.5. Instructions for the Design of the Blinding Device

#### 4.5.1. Guide Cane Shape Design

The overall black and white gray tone, simple and generous appearance, for the partially sighted groups does not need too much superfluous and decorative, taking into account the comfort and safety of the guide cane, streamlined design at the handle, and more closely fit the wrist area for flexible operation; cane body with a warning reflective coating, more visible in the dark, is not only to improve the sense of security of the blind themselves but also to protect the safety of these groups of travel. The pulley at the bottom of the cane automatically resets when the main body is magnetically charged, making it compact, flexible, and easy to operate. When the cane is combined with the charging post, it does not take up living space and is easy to store (see Figures 3–9).

In order to facilitate the travel of blind people, the charging post is usually placed in the corner of the entrance hall, making reasonable use of the corner space, and its both renewal functions, avoiding the problem of no socket.

By long pressing the red Braille button, Bluetooth connection with the guide device (cell phone and headset) is made, and the radar distance measurement at the bottom monitors the road conditions in real time to ensure normal and safe travel for the blind group. In case of emergency, the signal will be sent to the partially sighted group through the handle vibration and headphone alarm and the specific situation will be synchronized on the cell phone app of the family in time to improve the safety of the blind out (see Figures 10 and 11).

The article "Innovative Design of Intelligent Health Equipment for Helping the Blind in Smart City" was retracted in 2023. Reasons: signs of a paper mill; suspected computer-generated content; unreliable results or conclusions; concerns about the data.

#### 4.5.2. Guide Headset Design

The overall design of the headset consists of a headset charging case and a bone conduction headset to help the blind, and the headset case is placed in the groove of the crutch grip for wireless charging, while the headset is placed in the headset case can also be charged independently. The headset can work for 6–8 hours at full charge, and the headset charging case can be fully charged 4–5 times at full charge. Braille markings are set on the surface of the headset case to help blind people distinguish when picking it up.

Bone conduction headphones for the blind are designed in accordance with the principle of sound bone conduction, and the conductor is in the front of the outer ear, which can transmit sound through the skull to the hammer bone and can solve the problem of traditional headphones isolating the outside world and blocking the ear canal for too long to affect health and safety. The entire body of the headphones designed ear hooks can prevent the action amplitude is too large and drop the headphones, and ear hook shape is also based on the average ear position design, which can fit most people's ear shape, firmly fixed.

The overall color scheme of the headset box and headphones is mainly white and gray, and white is simple and generous, harmonious and elegant. The microphone is complemented by a distinctive, visible red so that some people with low vision can distinguish the wearing position, fashionable and beautiful, and good visual effect (see Figures 12–17).

#### 4.5.3. Guide Blind Software Page Design

This project uses a guide app, a smart guide stick, and a guide headset to interconnect things. All the designs in this project will be designed to achieve blind travel guidance for the visually impaired. The guide app exists to assist the visually impaired in their travels and to provide a degree of assistance that is necessary.

The functions of the guide software include basic information acquisition, blind and accessible path planning, and voice broadcasting. At present, the basic information for blind people to travel is mainly obtained by the existing map search and positioning functions. The blind and accessible path planning is to use the existing map navigation function to optimize the design of the walking path and to monitor the road conditions in real time during the walking process, so as to reduce the walking risk. The voice function is to provide voice prompts to blind people throughout the use process.

The guiding software is a kind of travel guidance structure for the blind with the guide stick and the guide headset as the core, which mainly assists the guide device to realize the functions of blind path guidance and timely risk avoidance.

The article "Innovative Design of Intelligent Health Equipment for Helping the Blind in Smart City" was retracted in 2023. Reasons: signs of a paper mill; suspected computer-generated content; unreliable results or conclusions; concerns about the data.

The project is a human-centered project that combines the idea of barrier-free design with the concept of universal design, and tries to explore a new, independent, and safe travel path based on the combination of the guide software and the guide device, breaking through the existing blind navigation system defects, efficiently avoiding the “broken head” and “snake” blindness. The project uses Bluetooth connection, handle vibration, and the ability to use the software.

The project uses Bluetooth connection, handle vibration, and other technologies to achieve voice navigation, GPS, and other functions for the user. The headset can be inserted in the groove of the handle for wireless charging.

In the process of traveling, the blind person first uses the guide app to voice input their destination, and the app uses the GPS map system for optimal path planning to calculate an optimal path for the blind person, and broadcast the direction in real time through the bone conduction headset for guidance. When starting to walk, some small obstacles that cannot be identified by the GPS system will require the radar function of the guide stick to alert in time, effectively avoiding obstacles and reducing the incidence of blind accidents. In case of emergencies that the blind cannot solve and handle by themselves, they can automatically contact their guardians and police through the one-touch alarm to avoid missing the best rescue time (see Figure 18).

## 5. Conclusion

During the course of this research, we researched the travel needs of the visually impaired group as well as the market for today's sight-aiding gadgets, combining and thoroughly analyzing the data of both to finish the design of this product. From the general concept, to the later details, to the physical design, to the final model, we went through a number of steps of proposing design ideas, determining, debugging, and optimizing. It provided us with a greater awareness of the societal relevance of blindness, as well as contemporary gadgets and apps for assisting the blind, as well as some regrets and concerns that may be discovered in the present study results. After conducting study for this project, I realized the difficulties that the blind face on a daily basis and recognized their need for a guide device. As a result, I met with the group members and the mentor to discuss the project's design for their safe trip, from the overall esthetic to the precise function design. However, there are some limitations in this design, such as the use of guide canes, guide headphones, and guide software; future devices for the blind require more depth; I hope to deepen my understanding of the blind through analysis and reflection, and further improve the devices for the blind so that the relevant people can accept them.

The article "Innovative Design of Intelligent Health Equipment for Helping the Blind in Smart City" was retracted in 2023. Reasons: signs of a paper mill; suspected computer-generated content; unreliable results or conclusions; concerns about the data.

## Figures and Tables

**Figure 1:** Existing smart glasses achievements.

**Figure 2:** Sketch of the concept and design of the intelligent blind guidance device.

**Figure 3:** The scheme determines the design.

**Figure 4:** Figure at the bottom of the guide stick.

**Figure 5:** Guide cane handle part diagram.

**Figure 6:** The structure of the blind cane is introduced and explained.

**Figure 7:** Front view of the guide stick.

**Figure 8:** Rear view.

**Figure 9:** Left view.

**Figure 10:** Use scene graphs.

**Figure 11:** Guided view of the blind person's travel.

**Figure 12:** Concept diagram of a guide headset.

**Figure 13:** Headset rendering.

**Figure 14:** Headset three views with dimensional drawings.

**Figure 15:** Braille identification.

**Figure 16:** Headphone structure explosion diagram.

**Figure 17:** Schematic of headset wearing.

**Figure 18:** Blind aid software interactive page design. (a) Look for the device page design. (b) Register the page design. (c) Map guide page design. (d) Radar obstacle avoidance reminder interface design.

## Data Availability

The dataset used to support the findings of this study is available from the corresponding author upon request.
